RETRACTED

# On the Innovation Mechanism and Communication Path of Philosophical Thinking in Innovative Community Environment

**DOI:** 10.1155/2022/7359420

**Published:** 2022-06-29

**Authors:** Xin Xin, Dayun Jiang

**Affiliations:** ^1^Jilin University, School of Philosophy and Society, Changchun 130012, Jilin, China; ^2^Jilin International Studies University, School of Marxism, Changchun 130017, Jilin, China

## Abstract

The development of philosophy has spawned a new type of interpersonal relationship, namely network community. As the main group of network applications, college students are an important part of the network community. Different from traditional thinking, community philosophical thinking has the remarkable characteristics of “equality, interaction, openness, and cooperation.” In the new media environment, we should fully learn from and learn philosophical thinking, carry out mechanism innovation, and form a “decentralized” network education community system; create a borderless network “education ecology”; build a network education model integrating “self-education” and “peer education”; promote the upgrading of network education mechanism from “one-way traffic” to “interactive participation”; and innovate the education mechanism in four aspects, so as to better meet the requirements of Education under the new media environment and improve the effect at the same time. Facing the era environment of philosophy and technology, the community environment should rely on the network community to study the innovation path. This paper first analyzes the connotation and characteristics of the online community, then discusses the innovation mechanism and communication significance of philosophical thinking based on the online community, and finally summarizes the innovation path of philosophical thinking based on the online community. By combing the impact and challenges brought by philosophy, this paper analyzes the necessity and importance of constructing innovation mechanisms under philosophical thinking, explains the rationality and superiority of innovation mechanisms under philosophical thinking, and puts forward some suggestions on constructing innovation mechanisms and communication path.

## 1. Introduction

Innovation is the main feature of the knowledge economy. The research scope includes organizational innovation, service innovation, management innovation, industrial innovation, and other fields. As a means of systematically studying the development law, dynamic mechanism, and performance of industrial innovation, the industrial innovation system has made a lot of achievements in recent years. With the advent of the era of philosophy, economic society has entered the field of a complex network. The actors in the economic system show strong nonlinear characteristics among each other. The interaction and closed-loop feedback of information and knowledge are highly important in modern technology represented by information technology [1]. Actors continue to learn from positive and negative feedback. The highly iterative technology has brought about great changes in the traditional mode of production, academic and scientific research cooperation [2]. In order to match the rapidly changing market environment and business model and pursue rapid access to the market, the traditional hierarchical management mode in technology-oriented enterprises is more changed to problem-solving or project team decision-making [3]. As a social system, the industrial innovation system is essentially a unified presentation of the patterned relationship network between different individuals and organizations. Therefore, it is feasible and necessary to study the industrial innovation system from the perspective of a network. The factors of different aggregates are different, and their goals and missions are also different. Only by truly mastering its connotation can it be innovated and spread. As shown in Table 1, with the development of philosophy and science and technology, online social networking has become the most commonly used way of people's communication. Online communities make the aggregation and dispersion of people's communication more flexible with interactivity, super space-time, freedom, and decentralization. An online community can highlight their personality elements and their value orientation [4]. Ideological and political education in Colleges and universities should rely on the network community, understand the communication methods of college students, grasp the ideological changes of college students, guide the mainstream thoughts of college students, and improve the effectiveness of ideological and political education in colleges and universities.

RETRACTED

Domestic research on Innovation based on complex networks includes small world characteristic innovation incubation network, industry-university research cooperation innovation complex network (Figure 1), the influence of interest-driven innovation network cooperation behavior evolution, the influence of a few large degree central nodes on the overall operational efficiency of complex networks, the innovation diffusion of complex networks under the influence of market orientation and multiagent cooperation, and so on. With the increase in technological complexity, a well-organized network has become the key to the success of innovation [5]. Promoting the self-organization of innovation networks and the decentralization of technology organizations are the key [6]. Johnsen and Ford studied collaborative innovation management in complex networks. Mccann et al. Constructed a multiparameter complex network innovation diffusion model, took the actor as the network node, and expressed the actor's adoption degree of innovation with variables, and the network node state was affected by the neighbor nodes [7].

## 2. Theory

### 2.1. Connotation and Characteristics of Online Community

The continuous development of philosophy and technology has led to the continuous emergence of various social software. People pay more and more attention to the sharing of topics in the process of online communication and will actively release information to attract more people's attention and resonate with others. The network-based communication group gathers with interest, keywords, personality, and other labels [8]. With the help of the network, the basic common interests or value orientation construct new relationships to form a network community, as shown in Figure 2.

The online community is a new type of relationship that individuals in the network gather spatially with the help of technology based on common values or interests [9]. The online community has the characteristics of the strong interaction, super time and space, high freedom, decentralization, and so on. The rise of online community takes the similarity of interest and emotion as the core, establishes an emotional connection through high-frequency interaction between groups, and then forms online ecological and cultural exchange [10]. Network community breaks through the limitation of traditional physical space and familiar circle and expands the communication space between people, with strong super space-time. The communication of an online community is based on freedom of speech, which blurs the identity of community members, so that the personality of members can be fully displayed. The communication of an online community is not centered on one person or one thing, but everyone is the center and everything is the center. It is a space world without a difference, which can effectively eliminate the discourse hegemony of traditional communication.

### 2.2. Research Progress of Online Community

Research on the virtual community at home and abroad has a long history [11]. In addition to the initial research on the definition, causes, nature, and characteristics of the virtual community, the research on customer innovation in the virtual community has become the focus of many scholars in recent years. Rheingold defined the concept of virtual community in 1993, which means that the virtual community is a number of people with the same emotional resonance and hobbies [12]. They communicate and exchange information with each other through a computer network. The existence of a computer network makes the connection between them get rid of the limitations of time and space. The virtual community itself also has great social and economic value [13].

RETRACTED

By combing the evolution of the concept of virtual community in China, Chinese scholars such as She Shuo (2018) once again defined the concept of virtual community with the help of bibliometric analysis tools and principles such as city space and excel and believed that the connotation of virtual community is a group that carries out centralized communication and interaction under certain conditions and has the same needs and interests, and its members have a strong sense of identity and trust [14]. In addition, through the research, we further clarify the differences between the virtual community and the virtual community in organizational structure and social attributes. The research systems of virtual community and open innovation are complete, but the degree of connection between theories is low [15]. The research on the virtual community at home and abroad has a long history and gradually forms a relatively complete system. The nature, characteristics, and functions of the virtual community have been gradually recognized by scholars. Although the research on open innovation started late, it is also relatively perfect in the aspects of concept definition, mode, realization way, and division of innovation resources [16]. Through the research already carried out by the above scholars, it can be found that the innovation resources from customer (user) groups have gradually become an important innovation element of product innovation in financial enterprises. However, after searching and combing the articles, it can be found that most of the existing research on the virtual community focus on the research on the internal fields of the virtual community, such as the definition, causes, and characteristics of the virtual community, which is relatively independent, and the collaborative research with other theories such as open innovation theory needs to be deepened, as shown in Figure 3.

### 2.3. Innovative Mechanism of Community Philosophical Thinking

The internal mechanism of philosophical thinking is an innovative mechanism in which the functions of reflection and sublation complement each other. The formation of this mechanism is a necessity for China's economic and social development [17]. Philosophical thinking and world outlook are interrelated and dialectically related, as shown in Table 2. Community is the product of the times, more precisely the product of the era of mobile philosophy. The development of mobile philosophy makes more mobile terminals become communication portals, forming decentralized communication. Since then, enterprises can have zero distance contact with users, which has brought great benefits to the promotion and sales of products [18]. Therefore, to be an enterprise, we must have community thinking. As far as the community itself is concerned, it is a new way of life and survival carrier of people in the era of mobile philosophy. It has constructed many new social relationships, and community thinking is based on this relationship. In fact, community thinking is circle thinking. The multiperson thinking mode mobilizes the collective wisdom and forms a powerful force. In addition, community thinking has also produced a new object relationship, that is, user thinking [19]. Therefore, there is no future without understanding community thinking. In the environment of community thinking, with the popularization of mobile philosophy, Internet access is everywhere, and the characteristics of mobile philosophy are brought into full play [20]. The first is zero distance; the second is decentralized propagation; and the third is the reorganization of distributed resources. These three factors lead to new changes and links in the relationship between people. These three kinds of links between people need to be maintained by action in order to realize their interaction, that is, community thinking. We know that the thinking mode of the traditional marketing model is to constantly tap new users without paying attention to the maintenance of old customers, resulting in the loss of old customers. Under this vicious circle, enterprises can only earn the middle difference to grow, and it is difficult to establish links with consumers.

RETRACTED

Chesbrough put forward the theory of open innovation in 2003. He believes that open innovation requires enterprises to break through closure, share and integrate internal and external innovation resources and technologies through external cooperation, and create value intensively. It is intended to improve the innovation ability of enterprises and realize a win-win for participants. It is a concept opposite to traditional closed innovation. Under the mode of open innovation, the innovation activities of enterprises will break through the limitations of traditional innovation subjects and no longer rely solely on internal forces. According to the division of resources, open innovation will make use of both internal and external innovation resources and internal and external commercialization resources. With the deepening of research, the status of customer groups, an important part of external resources, in enterprise open innovation has gradually attracted academic attention, and the important role of customer groups in participating in enterprise innovation has become increasingly clear. For example, piller (2003) specifically refers to the external innovation source of enterprise open innovation to the customer group and points out that open innovation is that enterprises collect and sort out various information from the customer group according to certain rules and then carry out activities such as product or service innovation, standard setting, and reinnovation.

Scholars define a cyber group as “a collection of digital individuals who take philosophy as the communication medium, take information connection as the link, seek mutual recognition due to common needs, and interact with social networks according to certain rules and methods.” Beyond the traditional limitations of blood, geography, and travel, online communities build a new type of interpersonal relationship of information and emotional communication for people of different genders, groups, and regions, guided by sharing, interaction, and social interaction. Relying on philosophy and technology, the development of the online community has experienced different stages and has become an important channel for people to obtain and share information. Web 1 stage: mainly portal forums represented by Sina, Sohu, Netease, Tencent, and People.cn. Massive information dissemination and interactivity began to appear, but they were not active. QQ group chat born during this period is mainly based on social attributes, and the attributes of media platforms have not been highlighted yet. Web2: in phase 0, web media such as forums, blogs, clients, microblogs, WeChat, and official accounts based on social functions have sprung up, and video sharing platforms such as iqiyi and Youku and webcast have emerged. During this period, the word “micro” came first, and the current development momentum is still strong. At this stage, the boundaries of the transmitting and receiving subjects are becoming increasingly blurred, and users often play multiple roles as information consumers, producers, and disseminators. Web3: stage 0 has begun to take shape. The intelligent ecology based on artificial intelligence, virtual reality, and big data makes the boundary between digital space and real life more blurred, even surreal.

The word “micro” stood out in the “2012 Chinese characters” selection sponsored by new weekly. In the selection of “2016 Chinese characters,” the word “brush” comes first. “Chinese inventory 2017” jointly sponsored by the national language resources monitoring and research center and the commercial press was elected. The Internet community has the characteristics of “decentralization, fragmentation, and fission,” which combines the characteristics of communication forms such as self-communication, interpersonal communication, organizational communication, and mass communication and integrates individuality, immediacy, and interactivity. The communication subject in the micro era has a diversified identity, democratized status, and decentralized power. The communication content is short and fragmented, which realizes cross-terminal and cross-platform aggregation, and conforms to the scene of people's fragmented consumption. The communication mode is mobile and visual, and the operation mode is simplified. Urban communication has realized the great migration from TV media to the philosophy field and from the replication of the PC terminal to the national creation of graphic and short videos on mobile terminals, which provides more new space and possibilities for urban “micro” communication.

RETRACTED

## 3. Necessity and Importance of Innovation Mechanism under Philosophical Thinking

### 3.1. Analysis on the Importance of Innovation Mechanism under Philosophical Thinking

College students are the fastest group to accept and praise new things. College students are active in the information age of mobile philosophy. To a certain extent, they have formed and widely used philosophical thinking to study and live. Respecting the characteristics of Internet thinking and making effective use of the advantages of philosophical thinking have important practical significance for the innovation mechanism.

#### 3.1.1. Innovation Mechanism under Philosophical Thinking Is the Dual Demand of Theoretical Research and Reality

In August 2014, Liu Qibao, director of the Propaganda Department of the CPC Central Committee, proposed to strengthen philosophical thinking and take mechanism innovation as the driving force. It can be seen that philosophical thinking has gradually become a bottom-up consensus, which will be fully reflected and applied in all fields of reform in China.

It is an important task for the construction of colleges and universities in China to adhere to building morality, cultivate people, and strengthen ideological guidance. The opinions on strengthening and improving the ideological and political work in Colleges and Universities under the new situation clearly puts forward that “establish philosophical thinking, promote the high integration of the traditional advantages of Ideological and political work and information technology, and make philosophy a new platform for ideological and political education.” Establishing philosophical thinking and exploring ideological and political education and talent training in colleges and universities under philosophical thinking are new topics that need to be solved urgently.

RETRACTED

#### 3.1.2. Definition of Philosophical Thinking and Innovation Mechanism

Philosophical thinking. What is philosophical thinking? There is no consensus in all walks of life. However, there is a consensus that it emphasizes “thinking,” which is a new way of thinking that uses the methods, rules, and spirit of philosophy to work, study, think, and live. It is not or not just a kind of technical thinking, marketing thinking, and e-commerce thinking, but a kind of systematic thinking, management thinking, and innovative thinking. It is realized through the platform of “philosophy.” There are different opinions on the characteristics of philosophical thinking, but they are inseparable from the obvious characteristics derived from philosophy, such as innovation, human nature, openness, convenience, equality, interaction, cooperation, and sharing. User thinking, platform thinking, dynamic thinking, social thinking, cross-border thinking, simple thinking, big data thinking, and iterative thinking are its basic attributes. Innovative mechanism. Mechanism refers to the structure, function, and relationship of organisms. The construction of a mechanism is a complex system engineering, including system and system. Education mechanism. It is an effective mechanism to explore the law of education management in Colleges and universities and the process of students' growth and success, stimulate the education function of each system through the interaction and coordination of various components of the ideological and political education system, form a joint force, and realize the purpose of education.

### 3.2. Analysis on the Necessity of Innovation Mechanism under Philosophical Thinking

#### 3.2.1. The Traditional Innovation Mechanism Cannot Meet the Needs of School Development and Student Growth in the New Era

Although the traditional innovation mechanism has the advantages of system inheritance and experience management, in the face of the higher education reform under the new normal, the traditional and invariable way of education gradually shows the disadvantages of emphasizing management over education, constraints over guidance, knowledge research over cultural shaping, and rule consciousness over ideology, as shown in Table 3. On the one hand, it is unable to keep up with the personality characteristics and growth needs of the “post-95” and “Post-00” young people who like fashion, pursue change, and are willing to accept new ideas and new things. In reality, they are keener on walking and using mobile philosophy, social networking, forums, and apps, which have become an indispensable part of their life and entertainment. They enjoy it anytime, anywhere, regardless of time and space. On the other hand, it cannot meet the requirements of building a world-class university and promoting the modernization of higher education. In order to deepen the reform and modernization of higher education, we must take building morality and cultivating people as the fundamental task of running a school. We must be more in line with the law of education and the law of talent growth, keep pace with the times, and constantly innovate, so as to build a modern education system with Chinese characteristics and realize the goal of “double first-class” construction and modernization of higher education.

RETRACTED

#### 3.2.2. Philosophy and New Media Have Brought New Impacts and Challenges to the Mechanism

Teaching. The traditional methods of theory teaching and assessment can no longer effectively achieve the effect of Ideological and political education, but what attracts students more are online learning, online discussion, online courses, and assessment. Therefore, the combination of MOCC, course sharing, flipped classrooms, online and offline hybrid teaching, examination system, and philosophy has begun to become the focus of teaching reform in colleges and universities.

Service. Students' access to information no longer only depends on posters and billboards but more on news and publicity released by public platforms. Therefore, apps and public platform numbers developed by various units came into being. Many news, notices, and news will be known to everyone in a very short time just by moving their thumb. All this benefits from philosophy.

Administration. In order to provide students with convenience without the time and place restrictions, save human and material resources, and realize students' daily management more efficiently, nowadays, students' payment, expenses, campus activities, dormitory occupancy, course selection, examination appointment, and other aspects of life, learning, and practice are also gradually connected by various professional systems or mobile app. All things on campus only need “online operation” or “card swiping.”

## 4. Strategies and Suggestions on the Communication Path of Online Community

The increasing reality of the online community provides a new opportunity for urban communication. For urban communication, the value of online community lies in the presentation and sharing of diversified, fragmented, refined, daily, and interesting urban information.

RETRACTED

### 4.1. Users: Both Content Production and Dissemination and Consumption

The emergence of the “Internet community,” a new type of social group, is of great significance in transforming the Internet in the sense of information technology into a social network in the sense of communication. In the online community, the threshold of information release is low, and the functions such as like, comment, forwarding, sharing, and collection are operated with one key, and the role of users as “messenger” is highlighted. Selfie, food, and scenic spots are hot topics, highlighting personal experience and a sense of existence. Online community communication tends to be sexual, interesting, and even fission. It inadvertently becomes famous overnight and has become a “punch in place” for popular tourism funds. The spread of celebrities in online communities cannot be underestimated. One sentence is often worth a thousand pounds, causing the fission effect (Figure 4), which is widely forwarded and discussed among fans, forums, and circles of friends.

The city image index and its test report issued by Zhejiang University United Technology Co. Ltd. actively affirmed the value of short videos in urban communication and comprehensively evaluated the effect of urban image communication from the four dimensions of popularity, breadth, depth, and potency. Among them, the popularity of communication mainly analyzes the urban communication power from five indicators: the number of users' creations, reading, likes, forwarding, and comments. Online communities have both user spontaneous production content (UGC) and professional production content (PGC).

High-quality development of new government media. The government actively guides with internet thinking, innovates communication methods and means, uses head-up attitude, and improves language style and narrative tone. It is becoming a high-quality content provider and leader in urban communication. Golden sentences appear one after another, brush the screen circle of friends, and become the norm. In March 2019, Hunan Changde Taohuayuan Cultural Tourism Festival opened. The secretary of the municipal party committee delivered a speech without writing. Using poetic language, he refined 11 “ones” to speak for Changde's “city in Taohuayuan,” which became a clear stream of government communication. Through online community forwarding, praise, and comments, the city image of “great beauty Changde” broke out instantly.

### 4.2. Short Video: The “Blue Ocean” of Urban Communication

According to the 43rd statistical report on China's Internet Development released by the China Internet Network Information Center (CNNIC), as of December 2018, the number of Internet users in China had reached 829 million, of which mobile Internet access accounted for 98.6%. The utilization rate of short video users is nearly 80%; the professionalism and verticality of content production are deepening; and high-quality content has become the core competitiveness of various platforms. It just confirms the evolution of the development model of China's online community from member aggregation to community brand and community economy. From the perspective of the audience's information acceptance, visual perception is more labor-saving and pleasant than words. In 2018, short videos represented by Tiktok and Kwai experienced a blowout, quickly surpassing the graphic mode and becoming a new “blue ocean” for urban communication. “Two micro and one shake” has become the standard configuration of urban image shaping and communication and has detonated the hot public opinion of the city from time to time. Government agencies have successively settled in microblogging, Tiktok, and other platforms and began to consciously carry out offline cooperation to achieve accurate communication. Xi'an Tourism Development Committee has reached comprehensive strategic cooperation with Tiktok to launch a full range of products based on Tiktok to promote Xi'an's cultural tourism resources. Small and medium-sized cities and towns “raised in the boudoir and unknown” used to be a blind spot for media communication, but they shine brightly in the community platform as shown in Figure 5.

RETRACTED

### 4.3. Media Platform: Social Operation

Media convergence is not only the direction of traditional media transformation but also the development opportunity of urban communication. Building an all-media communication pattern has become a national strategy. Therefore, urban communication should build “whole process media, holographic media, full member media, and full effect media”; comply with the social trend of community communication; and constantly expand and improve the communication power, guidance, influence, and credibility in cyberspace. “Changde, Hunan: the taste of civilization in the flexible morning market” is written in a small place, with a storytelling and strong human feelings. Seizing the “mobile morning market,” a scene of citizens' daily life, runs through the government's civilized city construction, which not only facilitates the lives of 30,000 residents around but also straightens out the relationship between urban management and hawkers, solves the problems of urban management so that people can obtain a real sense of happiness, and has a practical footnote to “ruling for the people.”

RETRACTED

The target of urban communication is people with different demands. It is required to establish user awareness and implement accurate communication. Community operation is an effective breakthrough path. There are three specific approaches: first, traditional media settle in various social platforms such as microblog and Tiktok, become a high-quality content provider of the platform with the help of traffic advantages, and realize the in-depth integration of traditional media content and social platforms, which is applicable to the grassroots local media with weak strength. Second, self-built all-media communication matrix. The news client of Hangzhou Daily puts forward the slogan “hang + hang family,” whose goal is to enter the families of ordinary citizens in Hangzhou. The “hang + school” launched by the group carries out community operation through segmentation, integrates educational resources, attaches great importance to community feedback, and realizes the benign operation of community content, users, values, business realization, and urban communication. Third, increase data-driven capacity-building. Integrate urban communication into the smart city construction system, share data resources, and achieve accurate communication.

## 5. Conclusion

With the rapid development of Internet technology, network social platforms emerge in endlessly, and network groups have become a new way for people to communicate. College students are the main force of network application, and the network community has become an important form of communication in their daily life and study. The openness and sharing of the online community make some philosophical thinking enter the vision of college students. Philosophical thinking guides college students through the platform of the online community. The innovation and dissemination of philosophical thinking based on the network community will help college students distinguish the ideology in the network community, broaden the work channels of Ideological and political educators in colleges and universities, enable college students to change the current situation of the object of traditional ideological and political education, and improve the effectiveness of Ideological and political education through active communication. The construction and dissemination of philosophical thinking based on an innovative network community can effectively stabilize ideology and enable college students to establish correct values.

## Figures and Tables

**Figure 1:** Schematic diagram of complex network relationship in the innovation community.

**Figure 2:** Classification of mainstream community networks.

RETRACTED

**Figure 3:** Research progress in an innovative community environment.

**Figure 4:** Fission form of community communication.

**Figure 5:** Top 10 players in Tiktok county.

**Table 1:** Comparative analysis of association and community/group/social network.

	Association	Community	Group	Social network
Leading factor	Manager LED	Manager LED	Manager LED	Individual led, no specific manager
Structure	Institutional centralization or decentralization structure	Institutional centralized structure	Centralized structure without system	Institutional decentralized structure
Goal and mission and opinion about value	Basic agreement	Values may be consistent, but goals and missions may be inconsistent	Have certain goals, but not necessarily mission and values	Completely inconsistent
Information transmission speed	Rapid	Slow	Rapid	Rapid

**Table 2:** Dialectical relationship between world outlook and philosophical thinking.

		World outlook	Philosophy
Difference	Meaning	People's general and fundamental views on the whole world	It is a theory about world outlook
	Subject	It is spontaneous; everyone has it	Through systematic learning, not everyone has it
	Characteristic	It is scattered and simple	Theoretical and systematic

Relation	The research object is the whole world. Philosophy is a systematic and theoretical world outlook. Philosophy takes the world outlook as its content and philosophy as its highest expression.		

**Table 3:** Scale and utilization rate of various community users in China (2020–2021).

Application	December 2020		December 2021		Growth rate (%)
	User scale (million)	Utilization rate of Internet users (%)	User scale (million)	Utilization rate of Internet users (%)	
Instant message	98,111	99.2	100,666	97.5	2.6
Online video (including short video)	92,677	93.7	97,471	94.5	5.2
Short video	87,335	88.3	93,415	90.5	7.0
Internet payment	85,434	86.4	90,363	87.6	5.8
Shopping online	78,241	79.1	84,210	81.6	7.6
Search engine	76,977	77.8	82,884	80.3	7.7
Networks news	74,274	75.1	77,109	74.7	3.8
Networks music	65,825	66.6	72,946	70.7	10.8
Networks broadcast	61,685	62.4	70,337	68.2	14
Online game	51,793	52.4	55,354	53.6	6.9
Online literature	46,013	46.5	50,159	48.6	9.0
Online takeout	41,883	42.3	54,416	52.7	29.9
Online car-hailing	36,528	36.9	45,261	43.97	23.9
Online office	34,560	34.9	46,884	45.4	35.7
Online travel booking	34,244	34.6	39,710	38.5	16.0
Online medical	21,480	21.7	29,788	28.9	38.7
Online investment products	16,988	17.2	19,427	18.8	14.4

## Data Availability

The labeled data set used to support the findings of this study is available from the corresponding author upon request.
